The article "Curcumin: the spicy modulator of breast carcinogenesis" was published in 2017. Journal: J Exp Clin Cancer Res.

# Curcumin: the spicy modulator of breast carcinogenesis

**DOI:** 10.1186/s13046-017-0566-5

**Published:** 2017-07-19

**Authors:** Urmila Banik, Subramani Parasuraman, Arun Kumar Adhikary, Nor Hayati Othman

**Affiliations:** 1 Department of Pathology, School of Medical Sciences, Universiti Sains Malaysia, 16150 Kubang Kerian, Kelantan Malaysia; 2 Unit of Pathology, AIMST University, Faculty of Medicine, Semeling, 08100 Bedong, Kedah Malaysia; 3 Unit of Pharmacology, AIMST University, Faculty of Pharmacy, Semeling, 08100 Bedong, Kedah Malaysia; 4 Unit of Microbiology, AIMST University, Faculty of Medicine, Semeling, 08100 Bedong, Kedah Malaysia

**Keywords:** Breast cancer, Carcinogenesis, Cancer hallmarks, Natural product, Curcumin

## Abstract

Worldwide breast cancer is the most common cancer in women. For many years clinicians and the researchers are examining and exploring various therapeutic modalities for breast cancer. Yet the disease has remained unconquered and the quest for cure is still going on. Present-day strategy of breast cancer therapy and prevention is either combination of a number of drugs or a drug that modulates multiple targets. In this regard natural products are now becoming significant options. Curcumin exemplifies a promising natural anticancer agent for this purpose. This review primarily underscores the modulatory effect of curcumin on the cancer hallmarks. The focus is its anticancer effect in the complex pathways of breast carcinogenesis. Curcumin modulates breast carcinogenesis through its effect on cell cycle and proliferation, apoptosis, senescence, cancer spread and angiogenesis. Largely the NFkB, PI3K/Akt/mTOR, MAPK and JAK/STAT are the key signaling pathways involved. The review also highlights the curcumin mediated modulation of tumor microenvironment, cancer immunity, breast cancer stem cells and cancer related miRNAs. Using curcumin as a therapeutic and preventive agent in breast cancer is perplexed by its diverse biological activity, much of which remains inexplicable. The information reviewed here should point toward potential scope of future curcumin research in breast cancer.

## Background

Breast cancer is the second most common cancer in the world accounting for 25% (approximately 1.67 million) of all new cancer cases diagnosed in 2012 [1]. It is the commonest cancer among women and levels as the fifth cause of death from cancer overall [2]. Although standard clinical practice requires screening and surveillance in the early detection of breast cancers, adherence to these guidelines is still low. Breast cancer thus far remains a lethal disease. For many years clinicians and researchers are examining and exploring various therapeutic modalities for breast cancer. Yet the disease has remained unconquered and the quest for cure is still going on.

The article "Curcumin: the spicy modulator of breast carcinogenesis" was published in 2017. Journal: J Exp Clin Cancer Res.

Cancer in breast commences in the terminal duct lobular unit (Fig. 1) and progresses in a stepwise manner [3]. It is a heterogeneous disease sustained by interconnected and intricate signaling pathways [4]. Diverse genetic and epigenetic alterations are crucial to this carcinogenesis [5, 6]. Thus aiming a single gene product or cell signaling pathway is unlikely to prevent or treat breast cancer. The current therapeutic options for breast cancer (surgical resection, radiation, and chemotherapeutic agents) [7–12] are not only costly but also modify many normal gene functions. Present-day strategy of breast cancer therapy and prevention is either combination of a number of drugs or a drug that modulates multiple targets. Nonetheless, it is still unknown how many cancer targets are there. Again how many targets must be confronted to control cancer growth is yet to be explored. In this regard natural products are now becoming significant option in breast cancer prevention and treatment. The well-known uses of these in cancer treatment are due to their effectiveness, less side effect, relatively low cost and notably their ability to target various signalling pathways. Thus they are the primary investigative molecules hovering hope of discovering new powerful classes of anticancer agents for breast cancer. One of the most noteworthy of these natural compounds is curcumin (diferuloylmethane). In the mid-eighties earliest investigations on the effect of curcumin revealed that it can be a potential anticancer agent [13, 14]. Subsequently researchers have been paying their attention to this unique compound. Cell type specific effects of curcumin are remarkable in selected cancers and only continued research can allow a better understanding of cell signaling pathways targeted by it.

**Fig. 1:** Schematic of segment of breast lobe showing the lobules and the duct system. The morphofunctional unit of breast is terminal duct lobular unit (TDLU). TDLU is a grapelike cluster of small alveoli that comprises lobule and terminal duct. The terminal ducts drains in to the subsegmental and segmental duct which drains into the lactiferous duct and collecting duct

Hallmarks of cancer encompass eight biological capabilities (sustaining proliferative signaling, escaping growth suppressors, resisting cell death, enabling replicative immortality, inducing angiogenesis, triggering invasion and metastasis, reprogramming of energy metabolism and evading immune destruction) acquired during cancer development [15]. Determining ways to suppress the transformed phenotypes can aid in advancement of new anticancer approach. The present review primarily focuses on the modulatory effect of curcumin on the cancer hallmarks and describes how the regulations can be applied practically in different anticancer approaches against this deadly disease. We also analyze the known impact of curcumin on microRNA and breast cancer stem cell (bCSC), two somewhat new areas of profound concern in cancer research.

The article "Curcumin: the spicy modulator of breast carcinogenesis" was published in 2017. Journal: J Exp Clin Cancer Res.

### What is curcumin and how it works?

Curcumin is a constituent of turmeric, the bright yellow spice, derived from the roots of plant *Curcuma longa* [3]. Turmeric is easily available, cheap and has a protracted history of being used as homemade remedies for different ailments. Chief component of the root is a volatile oil, containing turmerone. Curcuminoids are the coloring agents of turmeric. Curcuminoids consist of curcumin, demethoxycurcumin, 5′-methoxycurcumin, and dihydrocurcumin [3]. Curcumin (1,7-bis(4-hydroxy-3-methoxyphenyl)-1,6-heptadiene-3,5-dione), is a hydrophobic polyphenol (Fig. 2) [16]. It interacts with arsenals of molecules including inflammatory mediators, growth factors, enzymes, carrier proteins, metal ions, tumor suppressors, transcription factors, oncoproteins and cellular nucleic acids [17]. The interaction can be either indirectly or directly through covalent, non-covalent hydrophobic, and hydrogen bonding [18]. Its chemical structure with its different binding capacity is vital to its ability to interact with diverse targets. The reduced solubility and as a result lessened bioavailability is a recognized problem in the efficacy of curcumin. Solvents like dimethyl sulphoxide (DMSO), ethanol and sodium hydroxide are commonly used for dissolving curcumin. However studies showed that its solubility in water was significantly augmented with the application of heat [19, 20].

**Fig. 2:** The source and chemistry of curcumin. **a** Turmeric powder is obtained from the roots of plant *Curcuma longa.* **b** Curcumin is a component of turmeric. **c** The chemical structure of curcumin demonstrates a bis a, b-unsaturated diketone structure that displays keto enol tautomerism, with a predominant keto form in acidic and neutral solutions and a stable enol form in alkaline media. **d** The chemical structure of demethoxycurcumin and bisdemethoxycurcumin

The therapeutic properties of curcumin include antioxidant, antiarthritic, antiamyloid, anti-ischemic, and anti-inflammatory effect [21–23]. It has been shown to have protective and therapeutic efficacy against cancers of the skin, oral cavity, lung, pancreas, and intestinal tract, and to suppress tumor angiogenesis and metastasis [24–32]. Ever since the recognition of potential effect of curcumin on different cancer cells, different molecular studies have clarified its underlying mechanisms of actions in tumor cells. The multimodal targeting capacity of curcumin underlies its substantial therapeutic potential against cancer. Today we know that it exerts its anticancer effect by modulating different steps of multistep molecular carcinogenesis [33–36] (Fig. 3). This review will primarily focus and highlight how curcumin affects the cancer hallmarks.

The article "Curcumin: the spicy modulator of breast carcinogenesis" was published in 2017. Journal: J Exp Clin Cancer Res.

**Fig. 3:** Curcumin targets the different phases of carcinogenesis pathway. Curcumin affects the different phases of multistep molecular carcinogenesis. It modulates the cellular and molecular hallmarks of cancer and exerts its effects by affecting DNA mutations and epigenetic aberrations

### Curcumin and its growth inhibitory effect

The growth inhibitory effect of curcumin on breast cancer has been studied on different cancer models (Table 1). It impedes the growth of various cancer cells, without producing any toxicity to normal cells. Modulation of multiple cell signaling pathways that are linked with cell proliferation, cell cycle regulation, cellular senescence and apoptosis contribute in the process (Fig. 4).

**Table 1:** Growth inhibitory effect of curcumin on breast cancer

Effect	Curcumin alone or in combination	Model used (*cell line/**animal)	Expression phenotype of the cancer model	Solubilization of curcumin	Mechanism	Reference
Suppression of cell proliferation & cell cycle regulation	Curcumin	*MCF7	ER^+^ PR^+^ Her2^−^	Ethanol.	Inhibits phosphorylation of mTOR and its downstream effector molecule p70S6K and eukaryotic initiation factor 4E (eIF4E) binding protein 1 (4E-BP1),	[33]
	Curcumin	*MDA-MB-231 & BT-483	ER^−^ PR^−^ Her2^−^	Dimethyl sulphoxide (DMSO)	Down-regulation of NF-kB, cyclin D and MMP-1 transcription	[40]
	Curcumin	*Breast cancer cells BALB-neuT **BALB/c mice	Cancer cells expressing either high or low levels of ErbB2/neu.	Description not available	Down regulation of ERK1/ERK2 MAP kinases activity; dose dependant manner.	[43]
	Curcumin +Mitomycin C (MMC)	*MCF-7 **MCF-7 xenograft Female nu/nu athymic mice	ER^+^ PR^+^ Her2^−^	DMSO	p38 MAPK pathway mediated inhibition of cyclin D1, cyclin E, cyclin A, CDK2 & CDK4 with induction of cell cycle inhibitor p21, and p27.	[44]
	Curcumin	*MCF-7 & MDA-MB-231	ER^+^ PR^+^ Her2^−^ ER^−^ PR^−^ Her2^−^	DMSO	Inhibit expression of Wnt/β-catenin pathway components: disheveled, beta-catenin, cyclin D1 and slug with alteration of GSK3beta and E-cadherin.	[48]
	Curcumin	*MCF-7	ER^+^ PR^+^ Her2^−^	DMSO	Nrf2-mediated down-regulation of Fen1 expression; Nrf2 translocation from the cytoplasm to the nucleus and decrease Fen1 promoter activity by decreasing the recruitment of Nrf2 to the Fen1 promoter.	[51]
Apoptosis	Curcumin	*MCF-7	ER^+^ PR^+^ Her2^−^	Ethanol	Concentration-dependent regulation of genes related to cell death.	[53]
	Curcumin	*MCF 7, MDAH041 (post-crisis cell line from fibbroblasts of patient with LiFraumeni syndrome) & TR9-7 (derived from MDAH041 cells)	ER^+^ PR^+^ Her2^−^ MDAH041: the normal p53 allele has been lost during in vivo propagation. TR9-7: express wild-type p53 under control of tetracycline-regulated promoter	Description not available	Increase in p53 level & its DNA-binding activity followed by Bax expression at the protein level	[55]
	Curcumin	*ENU1564 (originated from an N-ethyl-N nitosourea-induced mammary adenocarcinoma in a female Berlin-Druckrey IV rat)		Description not available	Via intrinsic mitochondrial pathway; increased mitochondrial Ca (2+) and reactive oxygen species production with increased mitochondrial permeability transition.	[57]
	Curcumin	*MDA-MB-231	ER^−^ PR^−^ Her2^−^	DMSO	Dose-dependent inhibition of proliferation; increase Bax to Bcl-2 ratio; increases the protein level of p21 but decreases it for p53	[58]
	Curcumin +citral	*MCF 7	ER^+^ PR^+^ Her2^−^ ER^−^ PR^−^ Her2^−^	Description not available	Cell cycle arrest in G0/G1 phase; induced high levels of reactive oxygen species (ROS) generation and activated p53 and poly (ADP-ribose) polymerase-1 mediated apoptotic pathways.	[59]
	Curcumin	*MDA-MB-231	ER^−^ PR^−^ Her2^−^	Description not available	p53-Notch1 axis mediated downregulation of Notch1 and its downstream target, Hes1	[65]
	Curcumin	*MDA468 & HCC1806	ER^−^ PR^−^ Her2^−^	Ethanol	Induces double stranded DNA break in cancer cell; promotes phosphorylation of ATM/chk2-specific sites on BRCA1, total expression, and cytoplasmic retention of the BRCA1 protein; BRCA1 is retained in the cytoplasm where it cannot repair DNA damage; activates a DNA damage response in TNBC cells, leading to apoptosis	[68]
	Curcumin	*MCF-7	ER^+^ PR^+^ Her2^−^	DMSO	Suppression of IGF-1R gene expression; down-regulate the IGF-1 axis with a decrease in secretion of IGF-1 with a concomitant increase of IGFBP-3 in a dose-dependent manner.	[70]
	Curcumin	*MCF-7	ER^+^ PR^+^ Her2^−^	DMSO	Depolymerizes mitotic microtubules, disturbs microtubule-kinetochore attachment and the mitotic spindle structure. Activates the mitotic checkpoint and delays mitotic progression from metaphase to anaphase; p53 dependant apoptosis.	[71]
Induction of senescence	Curcumin+ silibin	*T47D	ER positive	DMSO	Decreases human telomerase reverse transcriptase (hTERT) gene expression	[73]
	Curcumin	*Patient-derived primary breast CAF cells (bCAF)		DMSO	p16-dependent, DNA damage independent; without associated inflammatory secretory phenotype	[74]

The article "Curcumin: the spicy modulator of breast carcinogenesis" was published in 2017. Journal: J Exp Clin Cancer Res.

**Fig. 4:** Targets in the curcumin mediated inhibition of breast tumor growth. Curcumin inhibits growth of breast cancer through inhibiting cancer cell proliferation, promoting apoptosis and inducing senescence by means of targeting multiple cell signaling pathways and transcription factors. NFκB: nuclear factor kappa B, MAPK: Mitogen-activated protein kinases, Wnt/β-catenin: Wingless-Int/beta-catenin, IGFR: Insulin like growth factor receptor, IGF1: Insulin like growth factor1, mTOR: mammalian target of rapamycin, ROS: reactive oxygen species, dsDNA: double stranded DNA, STAT3: Signal transducer and activator of transcription3, Nrf2: Nuclear factor (erythroid-derived 2)-like 2, hTERT: human telomerase reverse transcriptase

#### Modulation of cell proliferation and regulation of cell cycle

The growth and proliferation of cell is regulated by various interactions between the different molecules of cell cycle [37]. Multiple protein kinases control the major checkpoints in cell cycle and cyclin-dependent kinases (CDKs) and cyclins drive the cell through the cycle [38]. The expression of cyclins and CDKs are often aberrant in cancer cells and if these can be inhibited their transcription can be blocked and cell death can be induced. Thus currently the CDKs and cyclins are rational targets for cancer therapy [39]. Again constitutive activation of many signal transduction pathways also stimulate cancer cell growth. Besides there is crosstalk between these proliferative signaling pathways and the cell cycle regulators.

In breast cancer curcumin inhibits cell proliferation by down-regulating the transcription of nuclear factor kappa B (NF-κB), cyclin D and matrix metalloproteinase-1 (MMP-1) [40]. Curcumin can lead to cell cycle arrest both in G2/S and G2/M phase in different breast cancer cell lines, including the antiestrogen resistant ones [41, 42]. In CUR-treated cells the ERK (extracellular signal-regulated kinases)1/ERK2 mitogen-activated protein (MAP) kinases activity was down-regulated [43] and in combination with mitomycin C (MMC) there was enhanced G_1_ arrest with resultant inhibition of cancer cell proliferation and cycle progression in vitro and in vivo via the p38-MAPK pathway [44]. The antiproliferative effect of curcumin can also take place by means of AMPK(AMP-activated protein kinase) alpha-COX-2 pathway [45].

It is documented that abnormal activation of Wnt (Wingless-Int)/β-catenin signaling pathway and subsequent upregulation of β-catenin driven downstream targets c-MYC (Myelocytomatosis oncogene), and cyclin D1 is linked to breast carcinogenesis [46, 47]. Interestingly curcumin was found to inhibit the expression of various components of Wnt/β-catenin pathway including cyclinD1 in breast cancer cell line [48]. Again it is to be noted that curcumin’s growth suppressive action on estrogen receptor (ER) positive breast cancer cell is mediated through an ER related pathway and may interfere with 17- β estradiol at the receptor level [49].

The article "Curcumin: the spicy modulator of breast carcinogenesis" was published in 2017. Journal: J Exp Clin Cancer Res.

Flap endonuclease 1 (FEN1) represents a potent, broadly-applicable potential target for anticancer therapeutic development [50]. It is a DNA repair-specific nuclease and over-expression of FEN1 is involved in breast cancer development [50]. Curcumin may inhibit breast cancer cell proliferation through the transcription factor Nuclear factor (erythroid-derived 2)-like 2 (Nrf2) mediated down-regulation of Fen1 expression [51].

#### Induction of apoptosis

Apoptosis is a highly regulated mechanism by which cells undergo cell death. Inducing apoptosis in malignant cells without damaging normal cells is an effective but challenging anticancer approach. Curcumin has strong effect on both intrinsic and extrinsic pathways of apoptosis [52]. In breast cancer curcumin mediated apoptosis can take place through both p53 dependant and independent pathways.

Curcumin induced apoptosis in breast cancer cell is dose- and time-dependent and is regulated by multiple signaling pathways [43, 53, 54]. With curcumin treatment tumor-free survival was prolonged and tumor multiplicity was reduced in BALB-neuT mice [43]. It induced apoptosis via a p53-dependent pathway where Bax is the downstream effector [55, 56]. Curcumin alone or in combination with arabinogalactan promoted apoptosis by raising the ROS level, altering mitochondrial membrane and reducing glutathione [56]. Curcumin mediated induction of apoptosis by depletion of reduced glutathione has not been observed in breast cancer. It not only decreases the viability of murine mammary gland adenocarcinoma cell line by inhibiting Bcl-2 (B-cell lymphoma 2) and activating caspase-3, it increases mitochondrial Ca^2+^ and reactive oxygen species (ROS) production that act synergistically to produce the mitochondrial permeability transition and cell death [57]. It also induced apoptosis in breast cancer cells through up-regulating p21 expression [58]. Curcumin and citral combination treatment led to G0/G1 arrest in cell cycle. There was high levels of ROS generation only in breast cancer cells, which deactivated anti-apoptotic proteins like phosphorylated p53 and phosphorylated Bad and led to activation of apoptosis [59]. In combination with trichostin curcumin induces p53 independent apoptosis via c-Jun-N-terminal kinase (JNK) activation [60]. With berberine, curcumin induced caspase-dependent apoptosis in breast cancer cells via ERK (Extracellular Signal-regulated Kinase) pathways. Autophagic cell death was prompted through JNK (Jun N-terminal Kinase)/Bcl-2/Beclin1 pathway by this co-treatment [61]. Apoptosis is also induced in the breast cancer cells by curcumin mediated inhibition of intracellular fatty acid synthase expression [62].

The article "Curcumin: the spicy modulator of breast carcinogenesis" was published in 2017. Journal: J Exp Clin Cancer Res.

Notch gene family encodes evolutionarily conserved cell surface receptor. Overexpression of these receptors has been associated in breast cancer where Notch1 can be a transcriptional target of mutant p53 [63, 64]. Apoptosis in breast cancer cells can occur with abrogation of aberrant Notch1 signaling [64]. Treatment with curcumin resulted in downregulation of Notch1 and its downstream target, Hes1 due to the decreased activity of endogenous mutant p53 [65].

The tumor necrosis factor (TNF)- related-apoptosis-inducing ligand (TRAIL) is a potential anticancer agent, Once bound to the receptor, it leads to apoptosis by activating caspase-8 and downstream executioner caspases [66]. To normal cells TRAIL is pretty nontoxic. But it selectively fuels apoptosis in many transformed cells. Resistance is a major hurdle to the extensive use of TRAIL-based mono-therapies. Curcumin enhances TRAIL-induced apoptosis in breast cancer cells by regulating apoptosis-related proteins [67]. BRCA1 dysfunction is linked to triple negative breast cancer (TNBC) [68]. In TNBC cell lines curcumin induces double-strand breaks in DNA and increases expression as well as phosphorylation of DNA repair protein BRCA1. With cytoplasmic retention of BRCA1, DNA repair is hampered and cells undergo apoptosis [68]. Insulin like growth factors (IGFs) act as strong mitogens for a variety of cancer cells. The IGF-1 system has been implicated to play a critical role in breast carcinogenesis. This system comprises IGFs (IGF-1 and IGF-2), IGF-1 receptor (IGF-1R) and IGF binding proteins [69]. Curcumin suppresses IGF-1R gene expression at transcriptional level, down-regulates IGF-1 axis and blunts IGF-1-stimulated breast cancer cell growth and reverses the IGF-1-induced apoptosis resistance [70]. Curcumin lessens the microtubule instability of breast cancer cells, activates mitotic checkpoint, delays mitotic progression from the metaphase to anaphase and thus induces p53 dependent apoptosis [71].

#### Induction of senescence

Senescence is irreversible growth arrest. It prevents aged or abnormal cells from anarchic proliferation and is considered as a potent tumor-suppressing mechanism [72]. Telomere attrition and activation of tumour suppressor genes are two important mechanisms of cellular senescence. Telomere length is maintained by telomerase and progressive shortening of telomeres results in cell cycle arrest. In majority of breast cancer types telomerase is considerably activated [72]. Studies show that in breast cancer curcumin alone or in combination with silibin can inhibit telomerase expression [73]. It induces p16^INK4A^-dependent DNA damage-independent senescence without senescence associated secretory phenotype in breast cancer associated fibroblasts (bCAFs) [74].

The article "Curcumin: the spicy modulator of breast carcinogenesis" was published in 2017. Journal: J Exp Clin Cancer Res.

### Curcumin and its inhibition of cancer spread and tumor angiogenesis

For delivering oxygen and nutrients to the growing tumor, angiogenesis plays a key role. It is also critical for enabling two important malignant phenotypes: metabolic deregulation and tumor spread. As we know the degree of aggressive metastasis is an important prognostic factor for patients with breast cancer. Studies also suggests that metastasis may be an early event in the carcinogenesis process [75]. Once breast cancer has spread, treatment options are limited. Since most deaths from breast cancer occur after the disease has metastasized, inhibiting metastasis in the early phase of carcinogenesis is a potential therapeutic strategy against this cancer. Options to interfere with angiogenic signals by natural compounds with pleiotropic actions can be an alternative approach to develop a complementary anti-angiogenesis treatment strategy. Curcumin has effectively demonstrated its efficiency to act as a potent antiangiogenic, anti-invasive and anti-metastatic agent in vitro and in vivo in numerous occasions via modulation of mainly NF-κB, RhoA (Ras homolog gene family, member A)/ROCK (Rho-associated, coiled-coil-containing protein kinase 1)/MMPs and JAK2/STAT (Signal transducer and activator of transcription) 3 signaling pathway (Table 2).

**Table 2:** Curcumin mediated inhibition of breast cancer spread and angiogenesis

Effect	Curcumin alone or in combination	Model used (*cell line/**animal)	Expression phenotype of cancer cell	Solubilization of curcumin	Mechanism	Reference
Inhibition of invasion and metastasis	Curcumin	*MDA-MB-231 **Intercardiac injection of MDA-MB-231 cells in immunodeficient mice	ER^−^ PR^−^ Her2^−^	NaOH solution	Inhibits expression & activity of AP-1 & NFκB leading to diminished expression and activity of several MMPs; diminished IκB and p65 phosphorylation and reduced activation of the survival pathway NFκB significantly reduces the number of metastases.	[77]
	Curcumin	**MDA-MB-231 cells injected into the mammary fat pad of nude mice	ER^−^ PR^−^ Her2^−^	NaOH solution	prometastatic cytokines, CXCL1 & -2, which regulate the expression of CXCR4, the receptor for SDF1/CXCL12;	[78]
	Curcumin	*MCF-7 & MDA-MB-231	ER^+^ PR^+^ Her2^−^ ER^−^ PR^−^ Her2^−^	Description not available	ER-positive cancer: inhibits the expression of ER downstream genes including pS2 and TGF-beta and this inhibition is also dependent on the presence of estrogen ER negative cancer: reduced transcript levels of VEGF and b-FGF;b downregulated MMP-2 & upregulated TIMP-1	[49]
	Curcumin	*MDA-MB-435/β4 & MDA-MB-231	ER^−^ PR^−^ Her2^−^	Description not available	Reduced basal phosphorylation of beta(4) integrin; blocked alpha(6)beta(4)-dependent Akt activation and expression of cell motility-promoting factor ENPP2 (Ectonucleotide Pyrophosphatase/Phosphodiesterase 2).	[79]
	Curcumin	*MCF-7	ER^+^ PR^+^ Her2^−^	NaOH solution	Upregulated maspin expression with upregulation of p53 & downregulation of Bcl-2.	[81]
	Curcumin	*MCF-7	ER^+^ PR^+^ Her2^−^	Description not available	Concentration-dependent down regulation of RhoA and ROCK activities and expression of RhoA, ROCK1, ROCK2, MMP2 and MMP9; attenuation of RhoA/ROCK/MMPs pathway.	[82]
	Curcumin	*Patient-derived primary breast CAF cells (bCAFs)		DMSO	Inactivated the JAK2/STAT3 pathway; upregulated p16^INK4A^ & other tumor suppressor proteins; reduced the level of alpha-smooth muscle actin (α-SMA); suppressed the expression/secretion of stromal cell-derived factor-1 (SDF-1), IL-6, MMP-2, MMP-9, and TGF-β, which impeded their paracrine procarcinogenic potential; down-regulation of downstream targets c-Myc & survivin	[74]
	Curcumin	*MCF-7	ER^+^ PR^+^ Her2^−^	Description not available	Inhibition of PKCα-dependent MMP-expression, down- regulation of NF-κB and reduction of AP-1 activation; strongly repressed the TPA-induced phosphorylation of p38 and JNK and inhibited TPA-induced translocation of PKCα from the cytosol to the membrane.	[83]
	Curcumin	*MCF-7	ER^+^ PR^+^ Her2^−^	DMSO	Decreased the expression of uPA and NF-κB DNA binding activity,	[84]
	Curcumin	*MDA-MB-231, MDA-MB-468 & MCF-7	ER^−^ PR^−^ Her2^−^ (basal A and B) ER^+^ PR^+^ Her2^−^	Description not available	Down-regulates visfatin gene expression; decreased activity of constitutive NF-κB signalling.	[87]
	Curcumin	*MCF-7 & MDA-MB-231	ER^+^ PR^+^ Her2^−^ ER^−^ PR^−^ Her2^−^	Description not available	Down-regulation of LPS-induced markers of EMT such as vimentin via downregulation of NF-κB-Snail activity; upregulation of expression of E-cadherin	[95]
Inhibition of tumour angiogenesis	Curcumin	**MDA.MB231 xenograft model in Female Foxn1nu/nu mice	ER^−^ PR^−^ Her2^−^	Description not available	Inhibits activation of NF-*κ*B pathway with significant reductions in the expression of PECAM-1, cyclin D1, and p65;	[88]
	Curcumin	*MDA-MB-231	ER^−^ PR^−^ Her2^−^	Description not available	Inhibits OPN-induced VEGF expression by suppressing the binding activities of NF-κB & ATF-4.	[91]

Through down-regulation of NF-κBp65 expression and influencing its expression regulated gene products curcumin repressed tumor growth and microvessel formation in heterotopic breast cancer mouse model and inhibited migratory activity of cancer cells [58, 76]. It strongly averts the formation of hematogenous metastases in vivo through down-regulation of NF-κB/activator protein-1 (AP-1) dependent MMP expression and direct apoptotic effects on the circulating cancer cells [77]. Further study revealed that inhibition of NFκB reduced the expression of prometastatic chemokine (C-X-C Motif) ligand (CXCL)1 and −2, which in turn reduces expression of chemotactic receptor CXCR4 along with other prometastatic genes [78].

The article "Curcumin: the spicy modulator of breast carcinogenesis" was published in 2017. Journal: J Exp Clin Cancer Res.

While antiproliferative effects of curcumin are estrogen dependent in ER-positive human breast cancer cells, its anti-invasive effect on ER-negative cells was estrogen independent [49]. In the ER negative cancer while reducing the transcript levels of vascular endothelial growth factor (VEGF) and basic fibroblast growth factor, it downregulated MMP-2 and upregulated tissue inhibitor of metalloproteinase (TIMP-1). Integrin α_6_β_4_ is a laminin adhesion receptor linked to cancer cell invasion and migration. Akt and NF-κB are its known downstream effectors. Curcumin inhibits integrin function and blocks integrin-dependent breast cancer cell motility and invasion [79].

Maspin (mammary serpin) is a serine protease inhibitor. It can suppress tumor growth and metastasis in vivo and tumor cell motility and invasion in vitro. It links with the p53 tumor-suppressor pathway and functions as angiogenesis inhibitor both in vitro and in vivo [80]. Curcumin has shown to upregulate maspin expression in breast cancer cells [81]. While progressive loss of expression of maspin during tumor progression makes it a noteworthy biomarker, its curcumin mediated re-expression intervention offers a promising therapeutic option for breast cancer.

Lysophosphatidic acid (LPA) activates RhoA/ROCK/MMPs signaling pathway and induces as well as aggravates breast cancer invasion and metastasis. Curcumin inhibits LPA-induced cancer cell invasion by attenuating this pathway [82]. Activated cancer-associated fibroblasts or myofibroblasts facilitate tumor growth. Curcumin suppressed the procarcinogenic effects of stromal fibroblast [74]. It also repressed the 12-*O*-tetradecanoylphorbol-13-acetate (TPA)-induced MMP-9 expression and subsequent cell invasion [83]. It inhibited metastatic development via the suppression of urokinase- type plasminogen activator through NF-κB signaling pathways [84]. The association of breast cancer with obesity is linked to adipokines like visfatin [85, 86]. It was found that visfatin-Notch1 axis contributes to breast cancer progression [85]. Curcumin down-regulated the mRNA and protein levels of *visfatin* partly by NF-κB dependent mechanism [87].

The article "Curcumin: the spicy modulator of breast carcinogenesis" was published in 2017. Journal: J Exp Clin Cancer Res.

When treated with curcumin there was a substantial low level of expression of pro-angiogenic factors and a decrease in micro-vessel density in animals compared with that of vehicle treated tumors [88]. Curcumin revokes osteopontin (OPN) and progestin induced VEGF expression [89]. OPN upregulates expression of VEGF in human breast cancer model and pledges the angiogenesis [90, 91]. The chemokine-like extracellular matrix-associated protein OPN is pivotal in controlling breast cancer progression. Aiming the OPN-regulated signalling pathway by curcumin to turn off the angiogenic switch could be clinically valuable emergent tactic to the treatment of the disease.

With epithelial-mesenchymal transition (EMT) cancer cells attain molecular changes facilitating anomalous cell-cell adhesive interactions and junctions [92]. The cells morphologically become more spindle-shaped with subsequent loss of cell polarity and cell to cell adhesion [92]. This promotes cancer cell progression and spread. Once migrated to an appropriate location these cells upregulate epithelial markers through mesenchymal-epithelial transition. Subsequently there is activation of several transcriptional repressors through various vital signaling pathways like NF-κB, Wnt and Hedgehog [93, 94]. Therefore blocking or reversing EMT can be a promising anticancer strategy for restricting cancer spread. In breast cancer curcumin disrupts EMT and corresponding morphological changes with inhibition of cell motility and invasiveness in vitro [95]. It was also observed that curcumin decreased the expression of EMT related genes Slug, AXL and Twist1 in breast cancer cell lines [96].

### Curcumin and its impeding of cancer promoting inflammation

Chronic inflammation aids growth and spread of cancer through either direct interactions of inflammatory cells and cancer cells or indirect effects of inflammatory cells on other resident stromal cells. The cancer promoting effects of inflammation are release of growth factors, removal of growth suppressors, and enhanced resistance to cell death, initiation of angiogenesis, triggering of invasion and metastasis and evasion of immune destruction. Targeting the procarcinogenic products of inflammation like free radicals, arachidonic acid metabolites, NFκB transcription factor, TNF-alpha (TNF-α), CXC chemokines and AKT can be an important approach to halt cancer development and progression. Curcumin can inhibit iNOS (inducible nitric oxide synthase) induction, scavenge NO radicals in breast organ culture system and reduce free radical synthesis in the promotion phase of carcinogenesis [97, 98]. It can also downregulate CXC chemokines in via the NFκB pathway [78].

The article "Curcumin: the spicy modulator of breast carcinogenesis" was published in 2017. Journal: J Exp Clin Cancer Res.

Reprogramming of cellular energetic pathways in cancer cell is now a well-accepted fact which can be due to oncogene expression or inflammatory microenvironment [15, 99]. In cancer cells there is glucose amplified uptake and glycolysis. A substantial portion of glucose carbon from the augmented glycolytic catabolism is diverted to energize the cancer cell proliferation [100]. It was found that the inflammatory mediator TNF-α is a direct inducer of aerobic glycolysis and inhibitor of mitochondrial biosynthesis in malignant breast epithelial cell lines. Intriguingly this effect of TNF-α can be reversed by curcumin [101].

### Curcumin mediated modulation of breast cancer stem cells (bCSCs)

CSCs are tumor initiators and propagators of tumor growth. CD44 is an important cell surface markers for bCSCs. It is a downstream target gene of STAT3-NFκB signaling pathway. The spread of cancer is mediated by cellular component that displays high CD44 activity and is associated with an elevated level of microtentacles (McTNs) [102, 103]. McTNs aid in cell reattachment in the metastatic cascade. Alone or in combination with epigallocatechin gallate, curcumin blocked STAT3 phosphorylation, weakened the interaction between STAT3 and NFκB in the nucleus with downregulation of CD44 expression and resultant reduction in bCSC population [102]. Curcumin inhibited the bCSC subpopulation also by extinguishing McTNs [103]. Alone or in combination with piperine it is able to inhibit breast stem cell self-renewal through possible inhibition of Wnt signaling [104]. Moreover this combination downregulated stearoyl-coa desaturase, the regulator of stemness in breast stem cells [105]. This is clinically crucial as it can serve as an effective cancer preventing approach. A decreased expression of E-Cadherin, a transmembrane glycoprotein of cell adhesion, is associated with metastatic potential with poor prognosis in breast cancer. Breast CSCs are highly migratory cells. In these cells expression of E-cadherin is suppressed thus EMT is instigated. Curcumin amplifies the E-cadherin/β-catenin negative feedback loop and restores the expression of E-cadherin [106]. Hence this phytochemical can block bCSC migration and impede the EMT.

### Curcumin mediated modulation of tumor microenvironment and cancer immunity

The interplay between antitumor immunity and tumor-originated proinflammatory activity is thwarted in tumor microenvironment [15, 107]. Modulation of immune cells and the inflammatory process in order to manipulate the tumor microenvironment demonstrate attractive targets for therapeutic intervention in cancer. Again agents that can inhibit cancer-stroma crosstalk may augment conventional tumor cell directed therapy. It is recognised that exosomes secreted from the tumor cells fuses with the T cell and NK cell to supress their cytotoxicity and thereby promotes immune tolerance. In breast cancer curcumin can reverse this repression of NK cell cytotoxicity. In fact curcumin treatment enhances ubiquitination of exosomal proteins for degradation [108]. While curcumin has shown to have suppressive effect on bCAFs further study is looked-for to explore the effect of curcumin on the cross talks between cancer cell and stromal cells. Cutting-edge research should also focus on the immunomodulatory effects of this phytochemical on lymphoid cell populations, and cytokine production. Deeper understanding is needed as to whether it can be used alone or in combinations with different immunotherapies to therapeutic advantage.

The article "Curcumin: the spicy modulator of breast carcinogenesis" was published in 2017. Journal: J Exp Clin Cancer Res.

### Curcumin mediated modulation of cancer miRNA

Micro RNAs (miRNAs) are short non-coding RNA, each of which has the ability to regulate the expression of numerous genes. This feature allows them to simultaneously control multiple cellular signalling pathways. MiRNAs have been found to be dysregulated in nearly every types of human cancer including breast cancer [109, 110]**.** A slight change in the expression of one can generate a signaling cascade that has the potential to involve many molecular networks triggering various responses in cancer cell. Hence, miRNAs can be either targets or effectors. Since curcumin exerts its anticancer effects by targeting multiple signalling pathways, and miRNAs regulate diverse biological processes, it is thought that miRNAs could play a role in regulating response towards this natural agent (Fig. 5). This could lead to development of more effective treatment approaches. Whereas quite a few studies on various cancer demonstrated the anticancer effect of curcumin via modulation of miRNA, at present only few studies reveal curcumin-mediated miRNA regulation in breast cancer [109].

**Fig. 5:** Postulated aspects of curcumin mediated miRNA based modulation of breast cancer

Till now in breast cancer largely apoptosis, proliferation, invasion and metastasis have been found to be regulated by targeting miRNAs. In MCF-7 cells curcumin reduced Bcl-2 expression through upregulation of miR-15a and miR-16 and prompted cancer cell death [111]. Yet again when combined with emodin there was a synergism in its antiproliferative and anti-invasive effect through up-regulation of miR-34a [112]. As chronic inflammation promotes bystander cell survival with genomic injury it is a critical factor in the spread and growth of cancer. It has been found that curcumin up-regulates miR181b expression in metastatic breast cancer cells and directly binds to the 3′-UTR of CXCL-1 and -2. Subsequently there is down regulation of these proinflammatory cytokines. This up-regulation of miR181b inhibits metastases formation in vivo in immune-deficient mice [113]. The plastic derived universal chemical Bisphenol A (BPA) is an endocrine disrupter that has a cancer promoting effect in mammary epithelial cells. BPA mediates its carcinogenic effect via interference with miR-19 targeted PTEN/AKT/p53 axis with dysregulation of downstream proteins PTEN, p-AKT, p-MDM2, p53, and proliferating cell nuclear antigen. Fascinatingly curcumin restrained the upregulation of miR-19 and reversed cancer promoting effect of BPA [114].

The article "Curcumin: the spicy modulator of breast carcinogenesis" was published in 2017. Journal: J Exp Clin Cancer Res.

### Potential clinical implication of curcumin action

Curcumin exemplifies a promising natural anticancer agent for breast cancer prevention and treatment. All together the anticancer effect of curcumin mediated modulation of breast carcinogenesis is primarily through its impact on NFκB, PI3K/Akt/mTOR, MAPK, JAK2/STAT3 and Wnt/β-catenin signaling pathways (Fig. 6). The transcription factor STAT3 is constitutively activated in a major fraction of breast cancer types especially the estrogen negative types and TNBC [115]. Curcumin and its analogues have been found to inhibit cancer cell proliferation, promote apoptosis and suppress bCSCs by means of modulating this multifaceted transcription factor [102, 116, 117]. Curcumin is a good candidate for NFκB and STAT3 targeting. It may well represent a novel category of mTOR inhibitor and can also be an effective therapeutic agent in cancers with overexpression of integrin α_6_β_4_.

**Fig. 6:** Curcumin mediated modulation of major events in breast carcinogenesis. Curcumin exerts its anticancer effect by modulating cell proliferation and cell cycle regulation, inducing apoptosis and senescence, inhibiting cancer spread and tumor angiogenesis, impeding tumor promoting inflammation and modulating bCSCs, tumor microenvironment, cancer immunity and miRNA. bCSC: breast cancer stem cells, miRNA: microRNA, NFκB: nuclear factor kappa B, MAPK: Mitogen-activated protein kinases, mTOR: mammalian target of rapamycin, FeN1: Flap endonuclease 1, Nrf2: Nuclear factor (erythroid-derived 2)-like 2, Wnt/β-catenin: Wingless-Int/beta-catenin; IGF1: Insulin like growth factor1, CXCL: Chemokine (C-X-C Motif) Ligand, McTNs: microtentacles, VEGF: Vascular endothelial growth factor, RhoA: Ras homolog gene family, member A), ROCK: Rho-associated, coiled-coil-containing protein kinase 1), MMPs: Matrix metalloproteinase-1, bCAFs: breast cancer associated fibroblasts, JAK2/STAT3: Janus kinase 2/Signal transducer and activator of transcription3

Cancers have parenchymal and stromal component. Majority of the anticancer approach is primarily targeted towards the parenchymal part. However, CAFs comprise a major portion of the reactive tumor stroma. Hence efficient cancer therapy should take into account the presence of these stromal cells, which actively play a part in tumor growth and spread and may well be responsible for tumor recurrence. Curcumin might constitute an efficient fibroblast-directed therapeutic approach which may improve the outcome of classic therapeutic regimens of breast cancer.

The article "Curcumin: the spicy modulator of breast carcinogenesis" was published in 2017. Journal: J Exp Clin Cancer Res.

To date cytotoxic chemotherapy is the main therapeutic choice for TNBCs and with recurrence these cancers have no other treatment options. Curcumin-based treatment strategies may well improve the survival in patients with sporadic TNBCs. Last but not least, combining curcumin with chemo-based, hormone-based and targeted therapies can be a potential approach for the management of breast cancer.

## Conclusion

In breast cancer curcumin impedes tumor growth, malignant progression and spread. Usage of curcumin as a therapeutic agent in breast cancer is perplexed by its diverse biological activity, much of which remains unexplained. To conclude, along with the research for the enhancement of solubility and stability of curcumin, modulation of tumor microenvironment, cancer immunity, bCSCs, and cancer related miRNAs by this agent are important aspects where cutting-edge future study is looked-for.

## References

[1] Torre LA, Bray F, Siegel RL, Ferlay J, Lortet-Tieulent J, Jemal A (2015). Global cancer statistics, 2012. CA Cancer J Clin.

[2] Fact Sheets by Cancer. http://globocan.iarc.fr/Pages/fact_sheets_cancer.aspx. Accessed 7 Jan 2016.

[3] Sinha D, Biswas J, Sung B, Aggarwal BB, Bishayee A (2012). Chemopreventive and chemotherapeutic potential of curcumin in breast cancer. Curr Drug Targets.

[4] Singhal SK, Usmani N, Michiels S, Metzger-Filho O, Saini KS, Kovalchuk O (2015). Towards understanding the breast cancer epigenome: a comparison of genome-wide DNA methylation and gene expression data. Oncotarget.

[5] Khan SI, Aumsuwan P, Khan IA, Walker LA, Dasmahapatra AK (2012). Epigenetic events associated with breast cancer and their prevention by dietary components targeting the epigenome. Chem Res Toxicol.

[6] Parise CA, Bauer KR, Brown MM, Caggiano V (2009). Breast cancer subtypes as defined by the estrogen receptor (ER), progesterone receptor (PR), and the human epidermal growth factor receptor 2 (HER2) among women with invasive breast cancer in California, 1999-2004. Breast J.

The article "Curcumin: the spicy modulator of breast carcinogenesis" was published in 2017. Journal: J Exp Clin Cancer Res.

[7] Arslan C, Dizdar O, Altundag K (2014). Chemotherapy and biological treatment options in breast cancer patients with brain metastasis: an update. Expert Opin Pharmacother.

[8] Isakoff SJ (2010). Triple negative breast cancer: role of specific chemotherapy agents. Cancer J Sudbury Mass.

[9] Ishiba T, Nakagawa T, Sato T, Nagahara M, Oda G, Sugimoto H (2015). Efficiency of fluorodeoxyglucose positron emission tomography/computed tomography to predict prognosis in breast cancer patients received neoadjuvant chemotherapy. SpringerPlus.

[10] Shin SM, No HS, Vega RM, Fenton-Kerimian M, Maisonet O, Hitchen C, et al. Breast, chest wall, and nodal irradiation with prone set-up: results of a hypofractionated trial with a median follow-up of 35 months. Pract Radiat Oncol. 2015;10.1016/j.prro.2015.10.02226723552

[11] Shi Z, Peddi P, Burton G, Mills G, Shi R (2016). Effect of Postmastectomy radiation on survival of AJCC pN2/N3 breast cancer patients. Anticancer Res.

[12] van Rooijen JM, Stutvoet TS, Schröder CP, de Vries EGE (2015). Immunotherapeutic options on the horizon in breast cancer treatment. Pharmacol Ther.

[13] Jiang TL, Salmon SE, Liu RM (1983). Activity of camptothecin, harringtonin, cantharidin and curcumae in the human tumor stem cell assay. Eur J Cancer Clin Oncol.

[14] Kuttan R, Bhanumathy P, Nirmala K, George MC (1985). Potential anticancer activity of turmeric (*Curcuma longa*). Cancer Lett.

[15] Hanahan D, Weinberg RA (2011). Hallmarks of cancer: the next generation. Cell.

[16] Anand P, Sundaram C, Jhurani S, Kunnumakkara AB, Aggarwal BB (2008). Curcumin and cancer: an “old-age” disease with an “age-old” solution. Cancer Lett.

[17] Hasima N, Aggarwal BB (2012). Cancer-linked targets modulated by curcumin. Int J Biochem Mol Biol.

[18] Gupta SC, Prasad S, Kim JH, Patchva S, Webb LJ, Priyadarsini IK (2011). Multitargeting by curcumin as revealed by molecular interaction studies. Nat Prod Rep.

[19] Kurien BT, Singh A, Matsumoto H, Scofield RH (2007). Improving the solubility and pharmacological efficacy of curcumin by heat treatment. Assay Drug Dev Technol.

[20] Kurien BT, Harris VM, Quadri SMS, Coutinho-de Souza P, Cavett J, Moyer A (2015). Significantly reduced lymphadenopathy, salivary gland infiltrates and proteinuria in MRL-lpr/lpr mice treated with ultrasoluble curcumin/turmeric: increased survival with curcumin treatment. Lupus Sci Med.

[21] Bengmark S, Mesa MD, Gil A (2009). Plant-derived health: the effects of turmeric and curcuminoids. Nutr Hosp.

The article "Curcumin: the spicy modulator of breast carcinogenesis" was published in 2017. Journal: J Exp Clin Cancer Res.

[22] Jurenka JS (2009). Anti-inflammatory properties of curcumin, a major constituent of *Curcuma longa*: a review of preclinical and clinical research. Altern Med Rev J Clin Ther.

[23] Ringman JM, Frautschy SA, Cole GM, Masterman DL, Cummings JL (2005). A potential role of the curry spice curcumin in Alzheimer’s disease. Curr Alzheimer Res.

[24] Devassy JG, Nwachukwu ID, Jones PJH (2015). Curcumin and cancer: barriers to obtaining a health claim. Nutr Rev.

[25] Guo Y, Shu L, Zhang C, Su Z-Y, Kong A-NT (2015). Curcumin inhibits anchorage-independent growth of HT29 human colon cancer cells by targeting epigenetic restoration of the tumor suppressor gene DLEC1. Biochem Pharmacol.

[26] Jin H, Qiao F, Wang Y, Xu Y, Shang Y (2015). Curcumin inhibits cell proliferation and induces apoptosis of human non-small cell lung cancer cells through the upregulation of miR-192-5p and suppression of PI3K/Akt signaling pathway. Oncol Rep.

[27] Kim H, Park J, Tak K-H, Bu SY, Kim E (2014). Chemopreventive effects of curcumin on chemically induced mouse skin carcinogenesis in BK5.Insulin-like growth factor-1 transgenic mice. In Vitro Cell Dev Biol Anim.

[28] Lee AY-L, Fan C-C, Chen Y-A, Cheng C-W, Sung Y-J, Hsu C-P (2015). Curcumin inhibits invasiveness and epithelial-Mesenchymal transition in oral Squamous cell carcinoma through reducing matrix metalloproteinase 2, 9 and modulating p53-E-Cadherin pathway. Integr Cancer Ther.

[29] Liu L, Duan C, Ma Z, Xu G (2015). Curcumin inhibited rat colorectal carcinogenesis by activating PPAR-γ: an experimental study. Zhongguo Zhong Xi Yi Jie He Za Zhi.

[30] Wu J, Lu W-Y, Cui L-L (2015). Inhibitory effect of curcumin on invasion of skin squamous cell carcinoma A431 cells. Asian Pac J Cancer Prev.

[31] Wu L, Guo L, Liang Y, Liu X, Jiang L, Wang L (2015). Curcumin suppresses stem-like traits of lung cancer cells via inhibiting the JAK2/STAT3 signaling pathway. Oncol Rep.

[32] Zhao Z, Li C, Xi H, Gao Y, Xu D (2015). Curcumin induces apoptosis in pancreatic cancer cells through the induction of forkhead box O1 and inhibition of the PI3K/Akt pathway. Mol Med Rep.

[33] Beevers CS, Li F, Liu L, Huang S (2006). Curcumin inhibits the mammalian target of rapamycin-mediated signaling pathways in cancer cells. Int J Cancer J Int Cancer..

[34] Aggarwal BB, Kumar A, Bharti AC (2003). Anticancer potential of curcumin: preclinical and clinical studies. Anticancer Res.

[35] Kumar U, Sharma U, Rathi G (2017). Reversal of hypermethylation and reactivation of glutathione S-transferase pi 1 gene by curcumin in breast cancer cell line. Tumour Biol J Int Soc Oncodevelopmental Biol Med..

[36] Liu Y, Zhou J, Hu Y, Wang J, Yuan C (2017). Curcumin inhibits growth of human breast cancer cells through demethylation of DLC1 promoter. Mol Cell Biochem.

The article "Curcumin: the spicy modulator of breast carcinogenesis" was published in 2017. Journal: J Exp Clin Cancer Res.

[37] Choudhuri T, Pal S, Das T, Sa G (2005). Curcumin selectively induces apoptosis in deregulated cyclin D1-expressed cells at G2 phase of cell cycle in a p53-dependent manner. J Biol Chem.

[38] Hall M, Peters G (1996). Genetic alterations of cyclins, cyclin-dependent kinases, and Cdk inhibitors in human cancer. Adv Cancer Res.

[39] Dickson MA, Schwartz GK (2009). Development of cell-cycle inhibitors for cancer therapy. Curr Oncol.

[40] Liu Q, Loo WTY, Sze SCW, Tong Y (2009). Curcumin inhibits cell proliferation of MDA-MB-231 and BT-483 breast cancer cells mediated by down-regulation of NFkappaB, cyclinD and MMP-1 transcription. Phytomedicine Int J Phytother Phytopharm..

[41] Mehta K, Pantazis P, McQueen T, Aggarwal BB (1997). Antiproliferative effect of curcumin (diferuloylmethane) against human breast tumor cell lines. Anti-Cancer Drugs.

[42] Jiang M, Huang O, Zhang X, Xie Z, Shen A, Liu H (2013). Curcumin induces cell death and restores Tamoxifen sensitivity in the Antiestrogen-resistant breast cancer cell lines MCF-7/LCC2 and MCF-7/LCC9. Molecules.

[43] Masuelli L, Benvenuto M, Fantini M, Marzocchella L, Sacchetti P, Di Stefano E (2013). Curcumin induces apoptosis in breast cancer cell lines and delays the growth of mammary tumors in neu transgenic mice. J Biol Regul Homeost Agents.

[44] Zhou Q, Wang X, Liu X, Zhang H, Lu Y, Su S (2011). Curcumin enhanced antiproliferative effect of mitomycin C in human breast cancer MCF-7 cells in vitro and in vivo. Acta Pharmacol Sin.

[45] Lee YK, Lee WS, Hwang JT, Kwon DY, Surh YJ, Park OJ (2009). Curcumin exerts antidifferentiation effect through AMPKalpha-PPAR-gamma in 3T3-L1 adipocytes and antiproliferatory effect through AMPKalpha-COX-2 in cancer cells. J Agric Food Chem.

[46] Benhaj K, Akcali KC, Ozturk M (2006). Redundant expression of canonical Wnt ligands in human breast cancer cell lines. Oncol Rep.

[47] Mohammadi-Yeganeh S, Paryan M, Arefian E, Vasei M, Ghanbarian H, Mahdian R, et al. MicroRNA-340 inhibits the migration, invasion, and metastasis of breast cancer cells by targeting Wnt pathway. Tumour Biol J Int Soc Oncodevelopmental Biol Med. 2016;10.1007/s13277-015-4513-926758430

[48] Prasad CP, Rath G, Mathur S, Bhatnagar D, Ralhan R (2009). Potent growth suppressive activity of curcumin in human breast cancer cells: modulation of Wnt/beta-catenin signaling. Chem Biol Interact.

[49] Shao Z-M, Shen Z-Z, Liu C-H, Sartippour MR, Go VL, Heber D (2002). Curcumin exerts multiple suppressive effects on human breast carcinoma cells. Int J Cancer J Int Cancer.

The article "Curcumin: the spicy modulator of breast carcinogenesis" was published in 2017. Journal: J Exp Clin Cancer Res.

[50] van Pel DM, Barrett IJ, Shimizu Y, Sajesh BV, Guppy BJ, Pfeifer T, et al. An evolutionarily conserved synthetic lethal interaction network identifies FEN1 as a broad-Spectrum target for anticancer therapeutic development. PLoS Genet. 2013;9 doi:10.1371/journal.pgen.1003254.10.1371/journal.pgen.1003254PMC356105623382697

[51] Chen B, Zhang Y, Wang Y, Rao J, Jiang X, Xu Z (2014). Curcumin inhibits proliferation of breast cancer cells through Nrf2-mediated down-regulation of Fen1 expression. J Steroid Biochem Mol Biol.

[52] Elmore S (2007). Apoptosis: a review of programmed cell death. Toxicol Pathol.

[53] Ramachandran C, Rodriguez S, Ramachandran R, Raveendran Nair PK, Fonseca H, Khatib Z (2005). Expression profiles of apoptotic genes induced by curcumin in human breast cancer and mammary epithelial cell lines. Anticancer Res.

[54] Lv Z-D, Liu X-P, Zhao W-J, Dong Q, Li F-N, Wang H-B (2014). Curcumin induces apoptosis in breast cancer cells and inhibits tumor growth in vitro and in vivo. Int J Clin Exp Pathol.

[55] Choudhuri T, Pal S, Agwarwal ML, Das T, Sa G (2002). Curcumin induces apoptosis in human breast cancer cells through p53-dependent Bax induction. FEBS Lett.

[56] Moghtaderi H, Sepehri H, Attari F (2017). Combination of arabinogalactan and curcumin induces apoptosis in breast cancer cells in vitro and inhibits tumor growth via overexpression of p53 level in vivo. Biomed Pharmacother Biomedecine Pharmacother.

[57] Ibrahim A, El-Meligy A, Lungu G, Fetaih H, Dessouki A, Stoica G (2011). Curcumin induces apoptosis in a murine mammary gland adenocarcinoma cell line through the mitochondrial pathway. Eur J Pharmacol.

[58] Chiu T-L, Su C-C (2009). Curcumin inhibits proliferation and migration by increasing the Bax to Bcl-2 ratio and decreasing NF-kappaBp65 expression in breast cancer MDA-MB-231 cells. Int J Mol Med.

[59] Patel PB, Thakkar VR, Patel JS (2015). Cellular effect of Curcumin and Citral combination on breast cancer cells: induction of apoptosis and cell cycle arrest. J Breast Cancer.

[60] Yan G, Graham K, Lanza-Jacoby S (2013). Curcumin enhances the anticancer effects of trichostatin a in breast cancer cells. Mol Carcinog.

[61] Wang K, Zhang C, Bao J, Jia X, Liang Y, Wang X (2016). Synergistic chemopreventive effects of curcumin and berberine on human breast cancer cells through induction of apoptosis and autophagic cell death. Sci Rep.

[62] Fan H, Liang Y, Jiang B, Li X, Xun H, Sun J (2016). Curcumin inhibits intracellular fatty acid synthase and induces apoptosis in human breast cancer MDA-MB-231 cells. Oncol Rep.

[63] Lee CW, Raskett CM, Prudovsky I, Altieri DC (2008). Molecular dependence of estrogen receptor-negative breast cancer on a notch-Survivin signaling Axis. Cancer Res.

The article "Curcumin: the spicy modulator of breast carcinogenesis" was published in 2017. Journal: J Exp Clin Cancer Res.

[64] Simmons MJ, Serra R, Hermance N, Kelliher MA (2012). NOTCH1 inhibition in vivo results in mammary tumor regression and reduced mammary tumorsphere-forming activity in vitro. Breast Cancer Res BCR..

[65] Bae Y-H, Ryu JH, Park H-J, Kim KR, Wee H-J, Lee O-H (2013). Mutant p53-Notch1 signaling Axis is involved in Curcumin-induced apoptosis of breast cancer cells. Korean J Physiol Pharmacol.

[66] Garimella SV, Gehlhaus K, Dine JL, Pitt JJ, Grandin M, Chakka S (2014). Identification of novel molecular regulators of tumor necrosis factor-related apoptosis-inducing ligand (TRAIL)-induced apoptosis in breast cancer cells by RNAi screening. Breast Cancer Res.

[67] Park S, Cho DH, Andera L, Suh N, Kim I (2013). Curcumin enhances TRAIL-induced apoptosis of breast cancer cells by regulating apoptosis-related proteins. Mol Cell Biochem.

[68] Rowe DL, Ozbay T, O’Regan RM, Nahta R (2009). Modulation of the BRCA1 protein and induction of apoptosis in triple negative breast cancer cell lines by the Polyphenolic compound Curcumin. Breast Cancer Basic Clin Res.

[69] Singer C, Rasmussen A, Smith HS, Lippman ME, Lynch HT, Cullen KJ (1995). Malignant breast epithelium selects for insulin-like growth factor II expression in breast stroma: evidence for paracrine function. Cancer Res.

[70] Xia Y, Jin L, Zhang B, Xue H, Li Q, Xu Y (2007). The potentiation of curcumin on insulin-like growth factor-1 action in MCF-7 human breast carcinoma cells. Life Sci.

[71] Banerjee M, Singh P, Panda D (2010). Curcumin suppresses the dynamic instability of microtubules, activates the mitotic checkpoint and induces apoptosis in MCF-7 cells. FEBS J.

[72] Rodier F, Campisi J (2011). Four faces of cellular senescence. J Cell Biol.

[73] Nasiri M, Zarghami N, Koshki KN, Mollazadeh M, Moghaddam MP, Yamchi MR (2013). Curcumin and silibinin inhibit telomerase expression in T47D human breast cancer cells. Asian Pac J Cancer Prev.

[74] Hendrayani S-F, Al-Khalaf HH, Aboussekhra A (2013). Curcumin triggers p16-dependent senescence in active breast cancer-associated fibroblasts and suppresses their Paracrine Procarcinogenic effects. Neoplasia.

[75] Weng D, Penzner JH, Song B, Koido S, Calderwood SK, Gong J (2012). Metastasis is an early event in mouse mammary carcinomas and is associated with cells bearing stem cell markers. Breast Cancer Res.

[76] Bimonte S, Barbieri A, Palma G, Rea D, Luciano A, D’Aiuto M, et al. Dissecting the role of Curcumin in tumour growth and angiogenesis in mouse model of human breast cancer. Biomed Res Int. 2015;2015 doi:10.1155/2015/878134.10.1155/2015/878134PMC438656825879038

[77] Bachmeier B, Nerlich AG, Iancu CM, Cilli M, Schleicher E, Vené R (2007). The chemopreventive polyphenol Curcumin prevents hematogenous breast cancer metastases in immunodeficient mice. Cell Physiol Biochem Int J Exp Cell Physiol Biochem Pharmacol.

The article "Curcumin: the spicy modulator of breast carcinogenesis" was published in 2017. Journal: J Exp Clin Cancer Res.

[78] Bachmeier BE, Mohrenz IV, Mirisola V, Schleicher E, Romeo F, Höhneke C (2008). Curcumin downregulates the inflammatory cytokines CXCL1 and −2 in breast cancer cells via NFkappaB. Carcinogenesis.

[79] Kim HI, Huang H, Cheepala S, Huang S, Chung J (2008). Curcumin inhibition of Integrin (α6β4)-dependent breast cancer cell motility and invasion. Cancer Prev Res (Phila Pa).

[80] Maass N, Hojo T, Zhang M, Sager R, Jonat W, Nagasaki K (2000). Maspin--a novel protease inhibitor with tumor-suppressing activity in breast cancer. Acta Oncol Stockh Swed.

[81] Prasad CP, Rath G, Mathur S, Bhatnagar D, Ralhan R (2010). Expression analysis of maspin in invasive ductal carcinoma of breast and modulation of its expression by curcumin in breast cancer cell lines. Chem Biol Interact.

[82] Sun K, Duan X, Cai H, Liu X, Yang Y, Li M, et al. Curcumin inhibits LPA-induced invasion by attenuating RhoA/ROCK/MMPs pathway in MCF7 breast cancer cells. Clin Exp Med. 2015;10.1007/s10238-015-0336-725596714

[83] Kim J-M, Noh E-M, Kwon K-B, Kim J-S, You Y-O, Hwang J-K (2012). Curcumin suppresses the TPA-induced invasion through inhibition of PKCα-dependent MMP-expression in MCF-7 human breast cancer cells. Phytomedicine Int J Phytother Phytopharm.

[84] Zong H, Wang F, Fan Q-X, Wang L-X (2012). Curcumin inhibits metastatic progression of breast cancer cell through suppression of urokinase-type plasminogen activator by NF-kappa B signaling pathways. Mol Biol Rep.

[85] Park H-J, Kim S-R, Kim SS, Wee H-J, Bae M-K, Ryu MH (2014). Visfatin promotes cell and tumor growth by upregulating Notch1 in breast cancer. Oncotarget.

[86] Vona-Davis L, Rose DP (2007). Adipokines as endocrine, paracrine, and autocrine factors in breast cancer risk and progression. Endocr Relat Cancer.

[87] Kim S-R, Park H-J, Bae Y-H, Ahn S-C, Wee H-J, Yun I (2012). Curcumin down-regulates visfatin expression and inhibits breast cancer cell invasion. Endocrinology.

[88] Ferreira LC, Arbab AS, Jardim-Perassi BV, Borin TF, Varma NR, Iskander A, et al. Effect of curcumin on pro-angiogenic factors in the xenograft model of breast cancer. Anticancer Agents Med Chem. 2015;15:1285–96.10.2174/187152061566615052009364425991545

[89] Chakraborty G, Jain S, Kale S, Raja R, Kumar S, Mishra R (2008). Curcumin suppresses breast tumor angiogenesis by abrogating osteopontin-induced VEGF expression. Mol Med Rep.

[90] Carroll CE, Ellersieck MR, Hyder SM (2008). Curcumin inhibits MPA-induced secretion of VEGF from T47-D human breast cancer cells. Menopause.

The article "Curcumin: the spicy modulator of breast carcinogenesis" was published in 2017. Journal: J Exp Clin Cancer Res.

[91] Chakraborty G, Jain S, Kundu GC (2008). Osteopontin promotes vascular endothelial growth factor-dependent breast tumor growth and angiogenesis via autocrine and paracrine mechanisms. Cancer Res.

[92] Creighton CJ, Chang JC, Rosen JM (2010). Epithelial-Mesenchymal transition (EMT) in tumor-initiating cells and its clinical implications in breast cancer. J Mammary Gland Biol Neoplasia.

[93] Hardy KM, Booth BW, Hendrix MJC, Salomon DS, Strizzi L (2010). ErbB/EGF signaling and EMT in mammary development and breast cancer. J Mammary Gland Biol Neoplasia.

[94] Vuoriluoto K, Haugen H, Kiviluoto S, Mpindi J-P, Nevo J, Gjerdrum C (2011). Vimentin regulates EMT induction by slug and oncogenic H-Ras and migration by governing Axl expression in breast cancer. Oncogene.

[95] Huang T, Chen Z, Fang L (2013). Curcumin inhibits LPS-induced EMT through downregulation of NF-κB-snail signaling in breast cancer cells. Oncol Rep.

[96] Gallardo M, Calaf GM (2016). Curcumin inhibits invasive capabilities through epithelial mesenchymal transition in breast cancer cell lines. Int J Oncol.

[97] Onoda M, Inano H (2000). Effect of curcumin on the production of nitric oxide by cultured rat mammary gland. Nitric Oxide Biol Chem Off J Nitric Oxide Soc.

[98] Inano H, Onoda M, Inafuku N, Kubota M, Kamada Y, Osawa T (2000). Potent preventive action of curcumin on radiation-induced initiation of mammary tumorigenesis in rats. Carcinogenesis.

[99] Mauro C, Leow SC, Anso E, Rocha S, Thotakura AK, Tornatore L (2011). NF-κB controls energy homeostasis and metabolic adaptation by upregulating mitochondrial respiration. Nat Cell Biol.

[100] Lu J, Tan M, Cai Q (2015). The Warburg effect in tumor progression: mitochondrial oxidative metabolism as an anti-metastasis mechanism. Cancer Lett.

[101] Vaughan RA, Garcia-Smith R, Dorsey J, Griffith JK, Bisoffi M, Trujillo KA (2013). Tumor necrosis factor alpha induces Warburg-like metabolism and is reversed by anti-inflammatory curcumin in breast epithelial cells. Int J Cancer.

[102] Chung SS, Vadgama JV (2015). Curcumin and Epigallocatechin Gallate inhibit the cancer stem cell phenotype via down-regulation of STAT3–NFκB signaling. Anticancer Res.

[103] Charpentier MS, Whipple RA, Vitolo MI, Boggs AE, Slovic J, Thompson KN (2014). Curcumin targets breast cancer stem-like cells with microtentacles that persist in mammospheres and promote reattachment. Cancer Res.

[104] Kakarala M, Brenner DE, Khorkaya H, Cheng C, Tazi K, Ginestier C (2010). Targeting breast stem cells with the cancer preventive compounds Curcumin and Piperine. Breast Cancer Res Treat.

[105] Colacino JA, McDermott SP, Sartor MA, Wicha MS, Rozek LS (2016). Transcriptomic profiling of curcumin-treated human breast stem cells identifies a role for stearoyl-coa desaturase in breast cancer prevention. Breast Cancer Res Treat.

The article "Curcumin: the spicy modulator of breast carcinogenesis" was published in 2017. Journal: J Exp Clin Cancer Res.

[106] Mukherjee S, Mazumdar M, Chakraborty S, Manna A, Saha S, Khan P (2014). Curcumin inhibits breast cancer stem cell migration by amplifying the E-cadherin/β-catenin negative feedback loop. Stem Cell Res Ther.

[107] Casey SC, Amedei A, Aquilano K, Azmi AS, Benencia F, Bhakta D (2015). Cancer prevention and therapy through the modulation of the tumor microenvironment. Semin Cancer Biol.

[108] Zhang H-G, Kim H, Liu C, Yu S, Wang J, Grizzle WE (2007). Curcumin reverses breast tumor exosomes mediated immune suppression of NK cell tumor cytotoxicity. Biochim Biophys Acta.

[109] Iorio MV, Ferracin M, Liu C-G, Veronese A, Spizzo R, Sabbioni S (2005). MicroRNA gene expression deregulation in human breast cancer. Cancer Res.

[110] Di Leva G, Garofalo M, Croce CM (2014). microRNAs in cancer. Annu Rev Pathol.

[111] Yang J, Cao Y, Sun J, Zhang Y (2010). Curcumin reduces the expression of Bcl-2 by upregulating miR-15a and miR-16 in MCF-7 cells. Med Oncol.

[112] Guo J, Li W, Shi H, Xie X, Li L, Tang H (2013). Synergistic effects of curcumin with emodin against the proliferation and invasion of breast cancer cells through upregulation of miR-34a. Mol Cell Biochem.

[113] Kronski E, Fiori ME, Barbieri O, Astigiano S, Mirisola V, Killian PH (2014). miR181b is induced by the chemopreventive polyphenol curcumin and inhibits breast cancer metastasis via down-regulation of the inflammatory cytokines CXCL1 and −2. Mol Oncol.

[114] Li X, Xie W, Xie C, Huang C, Zhu J, Liang Z (2014). Curcumin modulates miR-19/PTEN/AKT/p53 axis to suppress bisphenol A-induced MCF-7 breast cancer cell proliferation. Phytother Res.

[115] Banerjee K, Resat H (2016). Constitutive activation of STAT3 in breast cancer cells: a review. Int J Cancer.

[116] Zhang X, Tian W, Cai X, Wang X, Dang W, Tang H (2013). Hydrazinocurcumin Encapsuled nanoparticles “re-educate” tumor-associated macrophages and exhibit anti-tumor effects on breast cancer following STAT3 suppression. PLoS One.

[117] Hutzen B, Friedman L, Sobo M, Lin L, Cen L, De Angelis S (2009). Curcumin analogue GO-Y030 inhibits STAT3 activity and cell growth in breast and pancreatic carcinomas. Int J Oncol.

